The article "Glycyrrhizic Acid Inhibits Core Fucosylation Modification Modulated EMT and Attenuates Bleomycin-Induced Pulmonary Fibrosis" was retracted in 2023. Reasons: signs of a paper mill; suspected computer-generated content; unreliable results or conclusions; concerns about the data.

# Glycyrrhizic Acid Inhibits Core Fucosylation Modification Modulated EMT and Attenuates Bleomycin-Induced Pulmonary Fibrosis

**DOI:** 10.1155/2022/5943322

**Published:** 2022-07-06

**Authors:** Lili Gao, Nan Wang, Yu Jiang, Jinying Hu, Baojie Ma, Taihua Wu

**Affiliations:** ^1^Department of Respiratory Medicine, The First Affiliated Hospital of Dalian Medical University, Dalian 116011, China; ^2^Department of Anesthesia, Dalian Women and Children's Medical Group, Dalian 116000, China

## Abstract

Idiopathic pulmonary fibrosis (IPF) is a fatal and incurable chronic interstitial lung disease with an unknown etiology. Recent evidence suggests that epithelial-mesenchymal transition (EMT) is one of the possible factors in the pathogenesis of pulmonary fibrosis. Glycyrrhizic acid (GA) is a natural active ingredient extracted from the root of the traditional Chinese herb licorice, which has been shown in previous studies to have the effect of alleviating lung injury. In this study, our objective was to investigate whether GA could ameliorate pulmonary fibrosis by altering EMT, as well as the therapeutic potential of changing core fucosylation (CF) to target EMT-related pathways. First, we verified that GA partially reverses EMT in a rat model of bleomycin-induced lung interstitial fibrosis, alleviating pulmonary fibrosis, and implying that GA has antifibrotic potential. Next, we discovered that GA attenuated lung interstitial fibrosis by reducing CF modifications to some extent. Interestingly, we found that GA therapy reduced the expression of phosphorylated Smad2/3 (p-Smad2/3) and *β*-catenin in the EMT pathway and that GA inhibited the modification of TGF-*β*R and WNT receptor proteins by CF, suggesting that GA may interfere with the EMT process by modulating TGF-*β*R, WNT core fucosylation modifications to attenuate pulmonary fibrosis. In conclusion, these findings indicate that GA could be a potential therapeutic agent for IPF, and further support the idea that targeting CF alterations could be a novel technique for the treatment of diseases involving EMT.

## 1. Introduction

Idiopathic pulmonary fibrosis (IPF) is an incurable and fatal chronic interstitial lung disease with a growing incidence and prevalence with age [1], and a survival period of 3–5 years after diagnosis [2]. The pathology of IPF is characterized by an enlarged interstitium with massive infiltration of inflammatory cells, thickening of the alveolar wall, and accumulation of extracellular matrix due to increased myofibroblasts, which eventually lead to the development of pathological fibrosis [3, 4]. Despite the fact that pirfenidone and nintedanib have been used in the clinic and have a good mitigation effect on IPF, there is still no conclusive evidence that these drugs can improve survival of patients [5, 6]. There are currently no effective treatments available to decrease the progression of lung interstitial fibrosis. As a result, it is critical to elucidate the potential development mechanism of pulmonary fibrosis, as well as to generate innovative intervention and therapy options.

The article "Glycyrrhizic Acid Inhibits Core Fucosylation Modification Modulated EMT and Attenuates Bleomycin-Induced Pulmonary Fibrosis" was retracted in 2023. Reasons: signs of a paper mill; suspected computer-generated content; unreliable results or conclusions; concerns about the data.

Epithelial-mesenchymal transformation is the process by which epithelial cells transform into mesenchymal cells, and it is an important aspect of developmental, wound healing, and other behaviors, along with pathologically promoting the advancement of fibrosis [7]. Lung epithelial cells have already been shown to develop into fibroblasts, and activated fibroblasts drive the formation of myofibroblasts while promoting the extracellular matrix. Fibrous tissue deposition and buildup gradually replace functional lung tissue, leading to structural failure of the lung parenchyma [8, 9]. Decreased expression of E-cadherin and increased expression of *α*-smooth muscle actin (*α*-SMA) in fibrosis models-induced by activation of bleomycin or TGF-*β* [4, 10, 11]. The signaling pathways that regulate EMT in the process of pulmonary fibrotic tissue injury and healing are complicated and diverse, and the TGF-*β*/Smad2/3 [12–14] and WNT/*β*-catenin signaling pathways [15–17] have been demonstrated to be intimately associated with EMT. As a result, a thorough understanding of the underlying processes of EMT, as well as the numerous molecular biological effects that may be generated by activation, is essential for developing effective treatments for IPF.

Glycosylation is a frequent posttranslational protein modification, which is necessary for many of the biological functions of glycoproteins [18]. Fucosyltransferase-catalyzed fucosylation is one of the most common types of glycosylation; *α*1,6-fucosyltransferase (FUT8) is the only enzyme in mammals that catalyzes core fucosylation (CF), and FUT8 catalyzes the transfer of fucosyl moiety to glycoproteins by forming *α*1,6 linkage, resulting in CF modifications [18, 19]. Significant progress has been made in the development of neoplastic disease diagnostic markers and medicines [20].

Licorice is one of the most popular legumes, according to the Chinese Pharmacopoeia, with a reddish brown or grayish brown surface, firm woody rhizome, and slightly fibrous cross section. Previous research has revealed that the phytoconstituents extracted from licorice include GA, isoliquiritin, glycyrrhizin, 18-glycyrrhetinic acid, glabrin A and B, liquiritigenin, and others [21]. These isolated metabolites have a wide range of biological properties, including antioxidant, anti-inflammatory, antiulcerative, antibacterial, immune-modulatory, and other activities [21–23]. Glycyrrhizic acid (GA) is a naturally extracted active ingredient from the roots of the traditional Chinese herbal medicine licorice. It is a part of triterpenoids, which are made up of two molecules of glucuronic acid and glycyrrhetinic acid, and are widely used as a sweetener in a variety of foods [24, 25]. In medicine, GA has been proven to inhibit lung cancer, leukemia, colon cancer, malignant glioma, and a variety of other cancers [26]. Furthermore, GA has been shown to reduce benzo(a)pyrene and LPS-induced lung damage [27, 28]. In addition, earlier research has shown that GA can suppress CCl4-induced apoptosis and liver fibrosis in rats [29]. Yet, its therapeutic effect and mechanism on bleomycin-induced pulmonary fibrosis in rats remain unknown. In this study, we found that GA can not only alleviate bleomycin-induced pulmonary fibrosis in in vivo but also inhibit the EMT process and the main mechanism may be related to the regulation of CF modification of TGF-*β*R and WNT, and affect the key protein in the TGF-*β*/Smad2/3 and WNT/*β*-catenin signaling pathways.

The article "Glycyrrhizic Acid Inhibits Core Fucosylation Modification Modulated EMT and Attenuates Bleomycin-Induced Pulmonary Fibrosis" was retracted in 2023. Reasons: signs of a paper mill; suspected computer-generated content; unreliable results or conclusions; concerns about the data.

## 2. Materials and Methods

### 2.1. The Rat Model of Pulmonary Fibrosis

8-weeks-old male specific pathogen-free (SPF) SD rats (240g-250 g, *n* = 40) from the Laboratory Animal Center of Dalian Medical University, they were kept at a constant temperature for a 12-hour light/dark cycle and were free to eat and drink. All experimental methods are carried out in accordance with guidelines formulated by the committee on the management and use of laboratory animals, and all animal experiments are carried out in accordance with procedures approved by the Laboratory Animal Ethics Committee of Dalian Medical University (AEE18071). Male SD rats were randomly divided into 5 groups, namely, the control group (*n* = 8), the fibrosis (BLM) group (*n* = 8), a 50 mg/kg GA treatment group (BLM + GA_50_, *n* = 8), a 100 mg/kg GA treatment group (BLM + GA_100_, *n* = 8), and a 200 mg/kg GA treatment group (BLM + GA_200_, *n* = 8). A single intratracheal injection of 5 mg/kg bleomycin (MB1039, Dalian Meilun, Dalian) or normal saline is given to the rats. Subsequently, the GA treatment group had to inject 50, 100, 200 mg/kg of GA (MB6163, Dalian Meilun, Dalian) intraperitoneally every day. At the same time, equal quantities of normal saline are injected into the abdominal cavity of the control and BLM group. After 4 weeks of intratracheal injection, all rats are killed. The upper lobe of the right lung is fixed in 4% paraformaldehyde solution, slices are histologically examined and the remaining right lobe and the left lung are cryopreserved at −80°C.

The article "Glycyrrhizic Acid Inhibits Core Fucosylation Modification Modulated EMT and Attenuates Bleomycin-Induced Pulmonary Fibrosis" was retracted in 2023. Reasons: signs of a paper mill; suspected computer-generated content; unreliable results or conclusions; concerns about the data.

### 2.2. Histopathological Examination

Lung tissue in fixed paraffin and slice it at 5 *μ*m. Slices were dewaxed with xylene I for 15 minutes, xylene II for 15 minutes, absolute ethanol I for 2 minutes, and absolute ethanol II for 2 minutes. After dewaxing, we perform H&E staining with hematoxylin concentrate (H8070, Solarbio, China) and eosin liquid (S23025101, Sinopharm, China), then we dehydrate with 80% ethanol, 90% ethanol, and absolute ethanol 1–2 s for three gradients of dehydration, then we transparent it with xylene I and xylene II for 2–3 s, and lastly, we seal it with neutral resin. Masson staining of dewaxed sections soaked in potassium dichromate solution for 20 min, followed by the same staining operation as above, then toluidine blue staining was soaked for 15 min, and finally dehydration, transparency, and sealing. Ashcroft scoring criteria were used to conduct a semiquantitative study.

### 2.3. Immunohistochemical Staining

The tissues are embedded in paraffin after fixation with 4% paraformaldehyde. The expression of collagen I and collagen III are detected by immunohistochemistry. Following the dewaxing wash, high-temperature antigen repair was performed with a citric acid antigen repair solution, followed by a 3% hydrogen peroxide endogenous peroxidase blocker (10011218, Sinopharm, China) for 10 minutes, a goat serum (SL2-10, Solarbio, China) block for 20 minutes, and overnight incubation with anti-collagen I antibody (Ab34710, ABCAM, USA) and anti-collagen III antibody (Ab7778, ABCAM, USA) at 4°C. Then, it was washed with PBS after 30 minutes at room temperature and incubated for 1 hour with the corresponding secondary antibody. The DAB color development kit is stained and observed under a microscope (DP73, OLUMPUS, Japan).

### 2.4. Western Blot

Lung tissue homogenate in lysate (P0013B, Beyotime, China) with protease inhibitors (ST506, Beyotime, China), centrifuged for 10 minutes at 4°C, 12000 rpm. The extracted supernatant is boiled and denatured after being treated with a 5 × loading buffer. Protein samples are separated by 10% SDS-PAGE electrophoresis, followed by protein transfer from gel to a PVDF membrane (IPVH00010, Millipore, USA). After 1 hour of blocking with 5% skim milk (Q/NYLB0039S, Yili, China), the membrane is incubated with the primary antibody overnight at 4°C. After three PBST washes of the membrane on the primary antibody, it is incubated for 2 hours at room temperature with the appropriate secondary antibody. Finally, the ECL kit (E002-5, Seven Seas Biology, China) was used to generate protein band pictures on the membrane. A semiquantitative study was conducted using an Image J software.

The article "Glycyrrhizic Acid Inhibits Core Fucosylation Modification Modulated EMT and Attenuates Bleomycin-Induced Pulmonary Fibrosis" was retracted in 2023. Reasons: signs of a paper mill; suspected computer-generated content; unreliable results or conclusions; concerns about the data.

### 2.5. Immunofluorescence

After fixation with 4% paraformaldehyde, tissues are paraffin-embedded. After the dewaxing wash, high-temperature antigen repair was performed with citric acid antigen repair solution, followed by 10 minutes with a 3% hydrogen peroxide endogenous peroxidase blocker, 20 minutes of blocking with goat serum, and overnight incubation with the primary antibody at 4°C. After 30 minutes at room temperature, it was washed with PBS and incubated for 1 hour with secondary antibodies. For 5 minutes, nuclei were stained with DAPI. Finally, using a laser confocal microscope, slices were examined and photographed.

### 2.6. Statistical Analysis

A GraphPad PRISM software (version 8.0; San Diego, CA, USA) was used to process the data, and the results are provided as the mean ± standard deviation (SD). To compare differences among various groups, one-way analysis of variance (ANOVA) was used, *T*-test was used for comparison between two groups. When *p* < 0.05, the differences are considered statistically significant.

## 3. Result

### 3.1. GA Alleviated Bleomycin-Induced Pulmonary Fibrosis in Rats

To investigate the impact of GA on reducing the severity of pulmonary fibrosis, we employed an in vivo model of bleomycin-induced pulmonary fibrosis in rats. After intratracheal bleomycin injection, a daily intraperitoneal treatment with different concentrations of GA is given. Compared to the control group, H&E and Masson staining revealed severe disruption of the structure of the lung section, collapse of the alveolar cavity, apparent thickening of the alveolar space, proliferation of a high number of fibroblasts, and accumulation of collagen fibers in lung tissue in the BLM group. In the GA treatment group, rat lung slices showed a more complete alveolar structure and a thinner alveolar wall, as well as a dose-dependent amelioration in bleomycin-induced collagen deposition (Figures 1(a) and 1(b)). Subsequently, compared to the BLM group, western blot analysis revealed that GA had a dose-dependent inhibitory effect on the expression of collagen I and collagen III in rat lung tissue (Figure 1(c)). Similarly, immunohistochemistry assays indicated that the expression of collagen I and collagen III in the GA treatment group was downregulated (Figure 1(d)). These results suggest that GA can alleviate the severity of bleomycin-induced pulmonary fibrosis to some extent.

### 3.2. GA Partially Reversed the Activation of EMT In Vivo

Next, we tried to confirm that GA can reduce the degree of bleomycin-induced lung interstitial fibrosis in rats by suppressing EMT. Therefore, we assessed the expression of E-cadherin, an alveolar epithelial cell marker, and *α*-SMA, a mesenchymal cell marker [10]. The expression of E-cadherin in the BLM group was significantly lower than in the control group, while the expression of *α*-SMA was significantly higher. In the GA treatment group, the expression of E-cadherin was higher than in the BLM group, while the expression of *α*-SMA was lower, suggesting that GA may intervene in the EMT process in IPF (Figure 2(a)). Consistent with this, immunofluorescence detection of lung tissue slices in rats further indicates that after treatment with GA, the expression of E-cadherin gradually extends with the increase of GA dose, *α*-SMA expression gradually weakened; the fluorescence intensity of E-cadherin in lung tissue in the high-dose GA treatment group was slightly lower, and the fluorescence intensity of *α*-SMA was slightly higher than that in the control group (Figure 2(b)). The above results strongly demonstrate that GA can modulate EMT in lung interstitial fibrosis and that the effect is dose-dependent.

The article "Glycyrrhizic Acid Inhibits Core Fucosylation Modification Modulated EMT and Attenuates Bleomycin-Induced Pulmonary Fibrosis" was retracted in 2023. Reasons: signs of a paper mill; suspected computer-generated content; unreliable results or conclusions; concerns about the data.

### 3.3. GA Inhibited CF Modification to Attenuate Pulmonary Fibrosis

Glycoproteomics studies have demonstrated that glycosylated modifications are required for glycoproteins to undergo translation and perform their biological activities [18, 30]. Protein glycosylation is essential in various ways, including spatial conformational folding, localization, and transport, as well as regulating receptor activation, and signaling channel transduction [31, 32]. To determine the effect of GA inhibiting CF modifications in rat lung interstitial fibrosis in in vivo, we examined the expression of FUT8. The expression of FUT8 in lung tissue decreased compared to the BLM group, which was associated with the GA dose. FUT8 expression in lung tissue was dramatically reduced as the GA dose increased, but the expression of FUT8 in lung tissue in the GA treatment group remained higher than in the control group (Figure 3(a)). In immunofluorescence staining, FUT8 was specifically recognized with green fluorescent markers and core fucose chain lectin FITC-LCA with red fluorescent markers, showing that normal rat lung tissues in the control group had moderate amounts of FUT8 and LCA expression, whereas FUT8 and LCA expression in lung tissues was dramatically elevated in the BLM group, and there was a positive correlation between FUT8 and LCA expression. Compared to the BLM group, the expression of FUT8 and LCA in lung tissue after treatment with GA decreased in a dose-dependent manner (Figure 3(b)). According to the findings, GA may regulate EMT-induced lung interstitial fibrosis in rats through CF modification, but it does not completely reverse the BLM-induced pulmonary fibrosis process.

The article "Glycyrrhizic Acid Inhibits Core Fucosylation Modification Modulated EMT and Attenuates Bleomycin-Induced Pulmonary Fibrosis" was retracted in 2023. Reasons: signs of a paper mill; suspected computer-generated content; unreliable results or conclusions; concerns about the data.

### 3.4. GA Inhibited the Expression of p-Smad2/3 and *β*-Catenin in EMT

GA activates a new signaling channel for prostate cancer that delays the EMT process [33]. Furthermore, the signaling mechanisms that control EMT during injury and healing of pulmonary fibrotic tissue are complicated and diverse, and the TGF-*β*/Smad2/3 [12–14] and WNT/*β*-catenin [15–17] pathways have been shown to be closely related to EMT. Based on the above findings, we investigate whether GA reduces pulmonary fibrosis by preventing the activation of critical proteins in EMT-related pathways. Western blot (Figure 4(a)) and immunofluorescence detection (Figure 4(b)) revealed that the expression of p-Smad2/3 was significantly higher in the BLM group compared to the control group, but gradually decreased as the therapeutic dose of GA increased, with significant differences between the high-dose GA group and the BLM group. Consistently, the expression of *β*-catenin was significantly higher in the BLM group than in the control group; in the GA treatment group, the expression of *β*-catenin in lung tissue gradually decreased and was dose-dependent, and the expression of *β*-catenin was still higher in the high-dose GA treatment group (Figure 4(c) and 4(d)). In conclusion, bleomycin-induced pulmonary fibrosis in rat models can activate the TGF-*β*/Smad2/3 and WNT/*β*-catenin pathways, and GA can have antifibrotic effects through the TGF-*β*/Smad2/3 and WNT/*β*-catenin pathways, although the change cannot be fully reversed. Interestingly, we did not find significant differences in Smad2/3 expression in rats' lung tissue in each group, which implies that TGF-*β*/Smad2/3 pathway activation is marked by Smad2/3 phosphorylation.

### 3.5. GA Inhibited the CF Modification of TGF-*β*R and WNT Receptor Protein

In previous research, FUT8 has been shown to be capable of CF modification of TGF-βRI on the surface of mouse lung tissue [34]. To further determine the changes of TGF-*β*R, WNT core glycosylation levels, and GA on the above receptor proteins and their CF modification levels in bleomycin-induced lung interstitial fibrosis, we applied an immunofluorescence staining assay to detect changes in CF modification of key receptor proteins in pathways related to bleomycin-induced pulmonary fibrosis. Detection by Western blot (Figure 5(a)) and immunofluorescence staining (Figures 5(b)–5(d)) suggests that compared with the BLM group, TGF-*β*RI, TGF-*β*RII, and WNT expression was elevated, the LCA content was significantly increased, and there were significant differences in the control group; in the GA treatment group compared to the BLM group, LCA expression decreased in a dose-dependent manner as GA concentration increased, and yet TGF-*β*RI, TGF-*β*RII, and WNT changes in the indicators are not significant. It was demonstrated that GA attenuated BLM-induced pulmonary fibrosis by regulating CF modifications of TGF-*β*RI, TGF-*β*RII, and WNT, important receptor proteins in the TGF-*β*/Smad2/3 and WNT/*β*-catenin signaling pathways, while having a little effect on the receptors themselves. Taken together, our findings support the view that GA mediates the antifibrotic effect by regulating EMT mainly through inhibition of TGF-*β*R and WNT core fucosylation modifications. As evidenced by the above findings, TGF-*β*RI, TGF-*β*RII, and WNT are all CF modified, and bleomycin-induced pulmonary fibrosis by upregulating CF modifications of TGF-*β*R and WNT receptors.

The article "Glycyrrhizic Acid Inhibits Core Fucosylation Modification Modulated EMT and Attenuates Bleomycin-Induced Pulmonary Fibrosis" was retracted in 2023. Reasons: signs of a paper mill; suspected computer-generated content; unreliable results or conclusions; concerns about the data.

## 4. Discussion

It is well known that the onset and evolution of pulmonary fibrosis is a complex process involving pathological processes, such as multiple signaling pathways. Our findings suggest that GA intervenes in EMT in pulmonary fibrosis and has a dose-dependent effect. In IPF, there are complex network systems for EMT-related signaling pathways [7, 9], and while previous research targeting solely upstream or downstream factors or receptors in a specific pathway was beneficial, escapes from activation of other signaling pathways invariably occurred. Therefore, common targets must be sought in a complex network of signal paths. Although the underlying molecular mechanism of IPF has not been elucidated, abnormal recapitulation of developmental lung gene expression, including TGF-*β* and WNT, has been linked to the abnormal wound healing process that occurs after repeated alveolar epithelial injury. TGF-*β* and WNT signaling are both involved in controlling cellular senescence and myofibroblast differentiation, cellular processes that have been considered as IPF treatment options [35–37]. Our study proved that bleomycin can induce activation of TGF-*β*/Smad2/3 and WNT/*β*-catenin pathways in rat pulmonary fibrosis models, and GA may have dose-dependent antifibrotic effects through the TGF-*β*/Smad2/3 and WNT/*β*-catenin pathways, but the change cannot be completely reversed. It is interesting to speculate about the role of CF modification in the pathology of IPF. According to our findings, FUT8 expression was significantly increased in rat pulmonary fibrosis models, demonstrating that CF modification can be activated to some extent during the pathogenesis of lung interstitial fibrosis. GA treatment can reverse CF activation in a dose-dependent manner. Previous studies have indicated that TGF- *β*R, a major receptor in the TGF-*β*/Smad2/3 pathway in renal interstitial fibrosis, can be modified with CF [38], while WNT, a receptor of the WNT/*β*-catenin pathway, is also a glycoprotein [39]. We reasonably hypothesize and demonstrate that major receptor proteins TGF-*β*R and WNT in the TGF-*β*/Smad2/3 and WNT/*β*-catenin signaling pathways can be modified by CF. GA inhibits CF modification as a means of antifibrosis and maintaining a balanced lung environment, helping to reduce bleomycin-induced pulmonary fibrosis.

The article "Glycyrrhizic Acid Inhibits Core Fucosylation Modification Modulated EMT and Attenuates Bleomycin-Induced Pulmonary Fibrosis" was retracted in 2023. Reasons: signs of a paper mill; suspected computer-generated content; unreliable results or conclusions; concerns about the data.

However, our current study has some restrictions. Due to experimental limitations, our study did not conduct in vitro experiments, and therefore could not more intuitively express the antifibrosis effect of GA. Furthermore, many drugs or active ingredients have previously been shown to be effective in animal models of bleomycin-induced pulmonary fibrosis but have not been effective in clinical trials [40]. This phenomenon merits further consideration and investigation. We hypothesize that a model of bleomycin-induced pulmonary fibrosis causes severe lung damage, despite the fact that the interstitial fibrosis phenotype is only a partial manifestation of lung injury and that this animal model does not represent all clinical features of human disease. As a result, to more strongly explain the therapeutic effect of GA on lung interstitial fibrosis, an animal model that is closer to clinical lung interstitial fibrosis must be established, such as transgenic animals [41].

Overall, our work is the first to discover the critical importance of CF modification in lung interstitial fibrosis, and GA intervened in EMT to attenuate pulmonary interstitial fibrosis by regulating the key receptor protein TGF-*β*R, WNT posttranslational CF modification, which elucidated the possible mechanism of GA for the treatment of IPF from a novel perspective and provided a new research direction for the clinical development of new drugs against pulmonary fibrosis. In addition, previous research [35, 42–44] discovered a crosstalk between the TGF-*β*/Smad2/3 and WNT/*β*-catenin signaling pathways. The WNT/*β*-catenin pathway stimulates the expression of TGF-*β* [45, 46], and TGF-*β* activates the WNT/*β*-catenin pathway [47, 48]. Our study also discovered that CF modifications can be a common target for these two pathways. Furthermore, it is also speculated that CF modification may serve as a link between pathways related to pulmonary fibrosis, paving the way for us to continue exploring the related mechanisms of pulmonary fibrosis centered on CF modification in the next step.

## 5. Conclusion

GA regulated EMT to attenuate BLM-induced pulmonary fibrosis by inhibiting CF modification of key receptor proteins TGF-*β*RI, TGF-*β*RII, and WNT in the TGF-*β*/Smad2/3 and WNT/*β*-catenin signaling pathway.

The article "Glycyrrhizic Acid Inhibits Core Fucosylation Modification Modulated EMT and Attenuates Bleomycin-Induced Pulmonary Fibrosis" was retracted in 2023. Reasons: signs of a paper mill; suspected computer-generated content; unreliable results or conclusions; concerns about the data.

## Figures and Tables

**Figure 1:** GA alleviated bleomycin-induced pulmonary fibrosis in rats. (a) Images of lung tissue stained with H&E. The scale bar is 200 *μ*m, and arrow points to the area with classic pulmonary fibrosis, which includes enormous fibroblast aggregation. (b) Images of lung tissue stained with Masson. The scale bar is 200 *μ*m, and arrow points to the area includes collagen deposition. (c) Western blot for the expression of Collagen I and III. (d) The expression of Collagen I and III in lung tissue detected by immunohistochemical staining. The scale bar is 200 *μ*m. ^*∗*^*p* < 0.05 vs. the control group; ^#^*p* < 0.05, ^##^*p* < 0.01, ^###^*p* < 0.001 vs. the BLM group.

**Figure 2:** GA partially reverses EMT activation in vivo. (a) Western blot was used to detect the expression of E-cadherin and *α*-SMA in the lung tissue of each group. (b) Images of immunofluorescence staining for E-cadherin and *α*-SMA. The scale bar is 200 *μ*m. ^*∗∗*^*p* < 0.01, ^*∗∗∗*^*p* < 0.001 vs. the control group; ^#^*p* < 0.05, ^##^*p* < 0.01, ^###^*p* < 0.001 vs. the BLM group.

**Figure 3:** GA inhibited CF modification to attenuate pulmonary fibrosis. (a) Western blot were used to detect the expression of FUT8. (b) Immunofluorescence staining for FUT8 and LCA in each group. The scale bar is 200 *μ*m. ^*∗∗∗*^*p* < 0.001 vs. the control group; ^##^*p* < 0.01, ^###^*p* < 0.001 vs. the BLM group.

**Figure 4:** GA inhibited the expression of p-Smad2/3 and *β*-catenin in EMT. (a) Western blot was used to detect the expression of Smad2/3 and p-Smad2/3 in the lung tissue of each group, followed by statistical analysis. (b) The immunofluorescence was used to detect the expression of p-Smad2/3. The scale bar is 200 *μ*m. (c) Western blot was used to detect the expression of *β*-catenin in the lung tissue of each group. (d) Immunofluorescence assay was used to detect the expression of *β*-catenin in the lung tissue of each group. The scale bar is 200 *μ*m. ^*∗∗∗*^*p* < 0.001 vs. the control group; ^##^*p* < 0.01, ^###^*p* < 0.001 vs. the BLM group.

**Figure 5:** GA inhibited the CF modification of TGF-*β*R and WNT receptor proteins. (a) Western blot was used to detect the expression of TGF-*β*RI, TGF-*β*RII, WNT, and LCA in the lung tissue of each group. (b)–(d) Immunofluorescence staining images of GA on TGF-*β*RI, TGF-*β*RII, WNT, and LCA expression. The scale bar is 200 *μ*m. ^*∗∗∗*^*p* < 0.001 vs. the control group; ^##^*p* < 0.01, ^###^*p* < 0.001 vs. the BLM group.

## Data Availability

The datasets generated and analyzed in this study are available from the corresponding author on reasonable request.
